# Internet+Continuous Nursing Mode in Home Nursing of Patients with T-Tube after Hepatolithiasis Surgery

**DOI:** 10.1155/2022/9490483

**Published:** 2022-05-31

**Authors:** You Peng, Huan Wan, Xiahong Hu, Fang Xiong, Yi Cao

**Affiliations:** ^1^The Second Department of Biliary Surgery, Hunan Provincial People's Hospital (The First Affiliated Hospital of Hunan Normal University), Changsha, 410000 Hunan, China; ^2^Department of Nursing, Hunan Provincial People's Hospital (The First Affiliated Hospital of Hunan Normal University), Changsha, 410000 Hunan, China; ^3^Department of Breast Armor Surgery, Hunan Provincial People's Hospital (The First Affiliated Hospital of Hunan Normal University), Changsha, 410000 Hunan, China

## Abstract

This study was to explore the effect of a continuous nursing model based on the mobile Internet in the home nursing of patients with T-tube after hepatolithiasis surgery. A continuous nursing system based on the mobile Internet was constructed, and 94 discharged patients with T-tube after biliary tract surgery were selected as the study subjects. The differences of complication rate, referral rate, nursing satisfaction, self-care ability, and quality of life score through the 36-item short form health survey (SF-36) after routine health education nursing (control group, *n* = 47) and continuous nursing mode based on the Internet (observation group, *n* = 47) were explored. The results showed that the success rate of the continuous nursing system based on mobile Internet in processing user requests was 96.2%. After nursing, the total complication rates of the control group and the observation group were 34.0% and 6.4%, the total satisfaction rates were 42.6% and 87.2%, and the referral rates were 23.4% and 6.4%, respectively, and the difference was statistically significant (*P* < 0.05). After nursing, the scores of self-care ability and SF-36 quality of life in the observation group were higher than those in the control group, and the difference was statistically significant (*P* < 0.05). In summary, the continuous nursing platform based on mobile Internet technology can meet the needs of users, and the nursing mode can significantly improve the home self-care ability of discharged patients with T-tube after surgery and improve the nursing effect, which is conducive to the rehabilitation of patients.

## 1. Introduction

Biliary tract disease is one of the most common diseases in hepatobiliary surgery, and patients undergoing biliary surgery usually require an indwelling T-tube in the common bile duct to remove residual stones [1]. T-tubes are generally placed for a long time, and maintaining smooth drainage and preventing shedding of T-tubes are very important to improve the therapeutic effect of patients [2, 3]. Generally, the tube is closed for 1 to 2 days after 10 to 14 days of T-tube drainage, and it can be removed without special circumstances, but some patients have underlying diseases, and the T-tube may be placed for one month or even longer in clinical practice. After discharge, patients should be closely observed for the patency of the T-tube, and improper care of discharged patients with T-tube will lead to different degrees of complications and even affect the prognosis of patients with severe conditions [4]. Therefore, there is a need to improve patients' self-care ability in home nursing, and hospitals usually achieve their goals through various health education programs [5]. The follow-up nursing platform built by medical institutions or personnel for discharged patients can provide continuous health services for patients, and the nursing model enables patients to receive professional nursing services during home rehabilitation [6]. Continuous nursing refers to extending nursing services from the hospital to the family or society and continuing the patient's rehabilitation status after discharge to meet the patient's needs [7]. The traditional method of nursing is health education for patients before discharge and continuous nursing by telephone interview [8]. However, the nursing effect of oral education is greatly affected by the knowledge level and acceptance ability of patients and their families, so only about 60% of the health training content can be remembered [9]. Telephone follow-up methods cannot directly observe the rehabilitation status of patients. If the patient's expressive ability is poor, it will also affect the follow-up effect [10].

The industries relying on Internet technology mainly include smart homes, smart transportation, and smart health care. Internet technology has changed the traditional form of medical treatment, and patients can flexibly choose the time and place to seek medical treatment, which greatly saves the treatment time and medical costs of patients and realizes the full use of resources [5]. The continuous nursing model based on Internet technology can effectively break through the limitations of region, time, and economy, realize the continuation from hospital to family/social care, optimize the health management of patients, enhance the self-management ability of patients, and meet the actual health needs [11]. For patients who perform home nursing, the continuous nursing platform constructed by Internet technology can enable patients to fully master nursing knowledge and conveniently, quickly, and interactively standardize their home nursing behavior [12, 13]. In addition, this model allows patients to contact medical staff at any time to improve the patient's care outcomes and prognosis [14]. At present, most of the Internet-based continuous nursing models are applied to home nursing for elderly patients or patients with chronic diseases, and there are relatively few studies on their application in the care of discharged patients with T-tube after hepatolithiasis surgery [15]. Therefore, the application effect of continuous nursing mode based on mobile Internet in home nursing of patients with T-tube after hepatolithiasis surgery was explored.

A continuous nursing platform based on Internet technology was constructed and applied to the continuous nursing of discharged patients with T-tube after hepatolithiasis surgery. The effects of nursing mode and routine health education on patients' rehabilitation effect, nursing satisfaction, self-care ability, and quality of life were compared, providing guidance and reference for improving the home nursing of patients with T-tube after hepatolithiasis surgery.

## 2. Research Methods

### 2.1. Mobile Internet System

The Android system is a very common mobile Internet technology, which is mainly applied to smart phones and mobile computers. It is an open-source mobile Internet operating system based on Linux. The basic framework of the Android system is shown in Figure 1. The Android system architecture is based on software stack, and the layers are separated from each other, and the division of labor is clear. The Android system is mainly composed of the application layer, application framework, function library, Android operation, and Linux kernel.

The core components of the Android system are activity, service, content provider, and broadcast receiver. Activity is the core and most common application component, and each interface of each application in the Android system can be regarded as activity. Service is similar to the basic functions of the activity, but the service does not have a visual interface, which runs mainly in the background to perform the background service or monitor the operation of the system. Content provider is one of the methods for data persistence in the Android system, and it is also the only method for supporting data sharing among different applications. Broadcast receiver is one of the mechanisms used in the Android system to process asynchronous message processing, which can be used to monitor or receive broadcasts sent by the system or application.

### 2.2. Design of Continuous Nursing System Based on Mobile Internet

The design of the mobile continuous nursing platform needs to be based on specific needs, including convenience. The data can be accurately uploaded to the remote server based on mobile Internet technology, so as to facilitate the medical staff to view the required information, thereby saving the time and energy of medical staff and patients, practicality and economy. There is almost no other cost after the installation of the mobile medical system, and the communication between patients and medical staff is conducive to the recovery of patients, scalability. In order to improve the function of the system, the system needs to add the function convenient for patients and medical staff, security. The system needs to use the algorithm to encrypt the patient data, so as to prevent the information from being leaked in the transmission process and ensure the privacy and security of patient information.

The constructed system is mainly composed of the operating system (CentOS6.5 system), application server (Web server), and database (MySQL database). The function of the system is given in Figure 2, which mainly includes the patient side, the manager side, and other functions. Each work side mainly refers to the patient information management, patient management, and health program management.

In order to verify the reliability of the system, different mobile phone clients were used to test the data of system server, and each functional process was detected in the system, so as to ensure that the system had no display and data transmission problems.

### 2.3. Study Subjects

The discharged patients with T-tube after biliary tract surgery in hospital from February 2019 to December 2021 were selected as the study subjects. There were 38 males and 56 females, aged 28-68 years old, with mean one of 48.9 ± 8.7 years old. Finally, 94 patients who met the requirements were included in the experiment and divided into the control group and the observation group according to the random number table, with 47 cases in each group. All patients signed the informed consent, and this study was approved by the ethics committee of hospital.

Inclusion criteria are as follows: patients undergoing biliary tract surgery after admission and indwelling T-tube more than 14 days; patients with normal cognitive function and no mental disorders; patients without heart, liver, kidney, and organic diseases of other important organs; patients and their families have electronic communication equipment capable of online communication; and patients who signed the informed consent.

Exclusion criteria are as follows: patients with serious postoperative complications, patients without electronic communication equipment for online communication, patients who cannot communicate normally, patients with cognitive dysfunction and mental disorders, and patients with malignant tumors, immune system abnormalities, or obvious organic organ lesions.

### 2.4. Nursing Methods

In the control group, the responsible nurse carried out routine discharge education according to the discharge instructions, including routine nursing of T-tube, dietary guidance, exercise mode guidance, medication guidance, lifestyle, and other precautions, and needed to observe the complications. The responsible nurse needed to give the patient or his/her family the contact information of the department and told the patient to return for examination in a timely manner in case of discomfort. A patient's personal electronic information file was constructed for follow-up in a telephone approach.

In the observation group, on the basis of routine care in the control group, the constructed Internet platform was used for continuous nursing of patients. Before patients were discharged from the hospital, a continuous nursing team with medical and nursing cooperation was established with the head nurse as the group leader, and full-time nurses were trained. A continuous nursing service manual and health education methods were developed. The questions of patients and their families were answered, and the mastery of “continuous nursing content” by patients' families was understood. Full-time nurses needed to make the content of health education as an electronic web page and uploaded it to the Internet continuous nursing platform every day, which included T-tube placement position and fixation method, observation of bile-related traits, treatment method of T-tube slippage, psychological counseling, diet, and medication guidance. The patient's family was given a contact method of the nurse on duty in order to cope with emergencies. Close communication with the patient's family and regular home visits were performed. Online and offline joint guidance for patients and their families was conducted to maintain the dry incision dressing; keep the surrounding skin clean; selection, fixation, and replacement of drainage bag; observation of bile color, quantity, and character changes; activity method carrying T-tube; drug use methods; and adverse reactions, and timely psychological counseling was carried out.

### 2.5. Observation and Evaluation Indicators

1. The basic data differences between the control group and the observation group were collected and compared, including the average age, sex ratio, education level, BMI, and other data of the control group and the observation group
2. Three different devices were selected for testing, and the number of samples was set to 200 to compare the success rate of continuous nursing system based on mobile Internet in processing user requests
3. The probability of complications such as pipeline blockage, pipeline shedding, infection, and bile leakage during nursing was recorded and compared, and the total incidence of complications was calculated
4. Comparison of nursing satisfaction: patient evaluation of nursing satisfaction. Satisfaction evaluation level was divided into dissatisfied, generally satisfied, satisfied, and very satisfied. Then, the total nursing satisfaction was calculated according to the equation: (the number of people who were very satisfied + the number of people who were satisfied)/total number × 100%
5. Comparison of referral rate: the probability of reexamination after discharge was recorded, and the reexamination rate was calculated according to the equation: the number of reexamination/total number × 100%
6. Patient self-care ability evaluation: during the period from carrying T-tube to extubation, the self-care ability of patients was evaluated using a self-made questionnaire. The design scale included dimensions such as dietary guidance, drug guidance, activity guidance, and psychological counseling, and each dimension scored 20 points. The total score of the scale was 100; the higher the score, the higher the patient's self-care ability
7. Quality of life evaluation: the 36-item short form health survey (SF-36) was used to evaluate the quality of life of patients. The scale contained eight dimensions to evaluate the health-related quality of life of patients, which were mainly divided into physical function (PF), role-physical (RP), bodily pain (BP), general health (GH), vitality (VT), social function (SF), role-emotional (RE), and mental health (MH). The higher the SF-36 score, the higher the quality of life of patients

## 3. Statistical Processing

Statistical analysis of the resulting data was performed using SPSS 19.0 software. Enumeration data were expressed as frequency (%), and chi-square test was used for difference analysis. Measurement data were expressed as mean ± standard deviation ($\bar{x}\pm s$), and independent sample *t*-test was used for difference analysis. *P* < 0.05 meant the difference was statistically significant.

## 4. Results

### 4.1. Continuous Nursing System Test Based on Mobile Internet

Three different devices were selected for testing, and the number of samples was set to 200 to compare the change in throughput, and the results are illustrated in Figure 3. The number of requests for this server to process data per minute was 4,887, while the success rate was approximately 96.2%. The concurrency of the platform can basically reach the requirements and can meet the needs of users.

### 4.2. Comparison of Basic Data of Patients

The differences in basic data between the control group and the observation group were collected and compared, and the results are shown in Table 1. There was no significant difference in the average age, gender ratio, education level, BMI, and other data between the control group and the observation group (*P* > 0.05).

### 4.3. Comparison of Incidences of Complications after Nursing

The differences in the probability of complications were recorded and compared, including pipeline blockage, pipeline shedding, infection, and bile leakage during nursing, and the total complication rate was calculated. The results are shown in Figure 4. The probability of pipeline blockage, pipeline shedding, infection, and bile leakage in the control group was 10.6%, 8.5%, 10.6%, and 4.3%, respectively. The probability of pipeline blockage, pipeline shedding, infection, and bile leakage in the observation group was 4.3%, 0.0%, 2.1%, and 0.0%, respectively. The total complication rates of the control group and the observation group were 34.0%, and 6.4%, respectively, and the difference was statistically significant (*P* < 0.05).

### 4.4. Comparison of Patient Satisfaction between the Two Groups after Nursing

Figure 5 shows the comparison of nursing satisfaction between the two groups of patients. The difference of satisfaction with nursing methods between the two groups was compared, and the total satisfaction rate was calculated. The probability of very satisfied, satisfied, generally satisfied, and unsatisfied in the control group was 23.4%, 19.1%, 19.1%, and 38.3%, respectively. The probability of very satisfied, satisfied, generally satisfied, and unsatisfied in the observation group was 61.7%, 25.5%, 4.3%, and 8.5%, respectively. The total satisfaction rates of the control group and the observation group were 42.6% and 87.2%, respectively, and the difference was statistically significant (*P* < 0.05).

### 4.5. Comparison of Referral Rate of Patients after Nursing

Figure 6 shows the difference in the referral rate and recurrence between the two groups. The differences in recurrence between the two groups during nursing were compared. The referral rates of the control group and the observation group were 23.4% and 6.4%, respectively, and the difference in the recurrence rate between the two groups was statistically significant (*P* < 0.05).

### 4.6. Comparison of Self-Care Ability after Nursing between the Two Groups

Figure 7 shows the comparison of self-care ability scores between the two groups. Differences in the self-care ability of patients after nursing were compared. After nursing, the scores of pipeline nursing, dietary guidance, drug guidance, activity guidance, psychological counseling, and the total average score in the self-care ability of patients in the observation group were higher than those in the control group, and the differences were statistically significant (*P* < 0.05).

### 4.7. Comparison of Quality of Life between the Two Groups after Nursing

Figure 8 suggests the comparison of quality of life scores between the two groups. Differences in quality of life of patients after nursing were compared. After nursing, the scores of PF, RP, BP, GH, VT, SF, RE, and MH in the observation group were higher than those in the control group, and the difference was statistically significant (*P* < 0.05).

## 5. Discussion

Intrahepatic and extrahepatic bile duct stones are very common diseases in hepatobiliary surgery, and surgical treatment is the main treatment method [16]. When intrahepatic and extrahepatic bile duct stones are treated surgically, the T-tube is usually placed in the common bile duct for drainage [17]. Indwelling T-tube can also achieve the purpose of bile drainage, bile duct support, and bile duct pressure reduction, thus reducing postoperative inflammation, edema, and bile outflow symptoms [18]. The time to carry T-tube after biliary surgery is about 10-14 days, and the indwelling time of patients with complex diseases will exceed 90 days [19]. With the gradual development of Internet science and technology, Internet medical care has become one of the effective ways to obtain high-quality health information services [20]. During hospitalization and discharge, only relying on health education of discharged patients with T-tube by medical staff cannot improve their mastery of T-tube management and nursing knowledge, thus affecting the prognosis of patients [21, 22]. The continuous nursing mode based on mobile Internet can ensure real-time communication between medical staff and patients; strengthen medical staff's grasp of patients' psychological problems, health management, and rehabilitation effect evaluation; and improve patients' trust in medical staff and patients' nursing satisfaction [23]. This nursing model can mobilize the subjective initiative of patients and their families, improve the self-care ability of patients and their families, and reduce the incidence of complications and referral rate in the nursing process [24]. The continuous nursing mode based on mobile Internet can shorten patients' return visit time, be conducive to postoperative rehabilitation, and ultimately improve patients' quality of life [25, 26].

In order to explore the nursing effect of continuous nursing model based on Internet technology for discharged patients with T-tube after hepatobiliary surgery, a continuous nursing platform based on mobile Internet was constructed and applied to home nursing for discharged patients with T-tube after hepatobiliary surgery, and the nursing effect was compared with traditional nursing. The results showed that the success rate of the continuous nursing system based on mobile Internet was about 96.2%, and the platform could basically meet the needs of users. The probabilities of pipeline blockage, pipeline shedding, infection, and bile leakage in the observation group were 4.3%, 0.0%, 2.1%, and 0.0%, respectively. The incidence rate of complications was 34.0% in the control group and 6.4% in the observation group. The total incidence rate of complications was significantly lower in the observation group, and the difference had statistical significance (*P* < 0.05). It revealed that the continuous nursing mode based on Internet technology can reduce the probability of complications in discharged patients with T-tube after hepatobiliary surgery, with higher safety. The total satisfaction rate of the control group and the observation group was 42.6% and 87.2%, respectively. The total satisfaction rate of the observation group was significantly higher than that of the control group, and the difference had statistical significance (*P* < 0.05). It can be observed that the continuous nursing mode was widely recognized by the patients, the acceptance rate was higher, and the effect was more significant. The referral rates of the control group and the observation group were 23.4% and 6.4%, respectively, which were significantly lower in the observation group than in the control group, and the difference had statistical significance (*P* < 0.05). After nursing, the scores of pipeline nursing, dietary guidance, drug guidance, activity guidance, psychological counseling score, and the total average score of self-care ability of patients in the observation group were higher than those in the control group, and the differences were statistically significant (*P*<0.05). After nursing, the scores of PF, RP, BP, GH, VT, SF, RE, and MH in the observation group were higher than those in the control group, and the differences were statistically significant (*P* < 0.05). The incidence rate of complications and follow-up rate of patients in continuous nursing mode based on mobile Internet were significantly lower than those of patients in routine nursing, and the self-care ability and quality of life scores of patients in continuous nursing mode were significantly higher than those of patients in routine nursing. It can be applied to home nursing of patients with T-tube after hepatolithiasis surgery and has positive application value.

## 6. Conclusion

A continuous nursing model based on Internet technology was proposed and applied to nursing of discharged patients. It was found that continuous nursing mode could reduce the incidence of complications and referral rate of discharged patients with T-tube and improve the nursing satisfaction, self-care ability, and quality of life of patients. The deficiency is that the sample size is too small to be further explored and proved.

## Figures and Tables

**Figure 1:** Basic architecture of mobile Internet (Android) system.

**Figure 2:** Functional framework of continuous nursing system.

**Figure 3:** Test results of continuous nursing system.

**Figure 4:** Comparison of the incidence of complications between the two groups. ^∗^Compared with the control group, *P* < 0.05.

**Figure 5:** Comparison of nursing satisfaction between the two groups. ^∗^Compared with the control group, *P* < 0.05.

**Figure 6:** Comparison of referral rate between the two groups. ^∗^Compared with control group, *P* < 0.05.

**Figure 7:** Comparison of self-care ability scores between the two groups. ^∗^Compared with the control group, *P* < 0.05.

**Figure 8:** Comparison of quality of life scores of patients. ^∗^The difference between groups was statistically significant, *P* < 0.05.

**Table 1:** Comparison of basic data of patients.

Basic data	Control group (*n* = 47)	Observation group (*n* = 47)	*t* or *χ*^2^	*P*
Age (years old)	43.9 ± 4.5	44.8 ± 5.5	-0.339	0.243
Gender (*n* (%))			0.417	0.305
Male	18 (19.1)	20 (21.3)		
Female	29 (30.9)	27 (28.7)		
Cultural level (*n* (%))			0.126	0.414
Primary school and below	8 (8.5)	10 (21.3)		
Middle school	23 (24.5)	26 (27.7)		
College and above	16 (17.0)	11 (11.7)		
BMI (kg/m^2^)	21.8 ± 2.1	22.2 ± 3.7	0.191	0.155

## Data Availability

The data used to support the findings of this study are available from the corresponding author upon request.
